# SDR9C7 Promotes Lymph Node Metastases in Patients with Esophageal Squamous Cell Carcinoma

**DOI:** 10.1371/journal.pone.0052184

**Published:** 2013-01-14

**Authors:** Shanhong Tang, Liucun Gao, Qian Bi, Guanghui Xu, Simeng Wang, Guohong Zhao, Zheng Chen, Xiushan Zheng, Yanglin Pan, Lina Zhao, Jianqin Kang, Guitao Yang, Yongquan Shi, Kaichun Wu, Taiqian Gong, Daiming Fan

**Affiliations:** 1 State Key Laboratory of Cancer Biology, Xijing Hospital of Digestive Diseases, Fourth Military Medical University, Xi’an, People′s Republic of China; 2 Department of Thoracic Surgery, Daping Hospital, Third Military Medical University, Chongqing, People′s Republic of China; INRS, Canada

## Abstract

**Background:**

The major reason for the poor prognosis of esophageal squamous cell carcinoma (ESCC) patients is lymph node (LN) metastases.

**Methodology/Principal:**

In the present study, gene expression profiling assay (GEP) was performed to identify the differences in gene expression profiles between primary ESCC tumors that were with LN metastases (N_+_) and those without LN metastases (N_-_).

**Conclusions/Significance:**

A total of 23 genes were identified as being significantly elevated, and 30 genes were sharply decreased in ESCC tumors that were N_+_ compared with N- tumors. Among these genes, two transcripts of the short chain dehydrogenase/reductase family 9C, member 7 (SDR9C7) were observed 7 times more frequently in N_+_ compared with N_-_ tumors. Immunohistochemical staining showed that SDR9C7 expression closely correlated with metastasis, and would be a prognostic marker for ESCC patients. To investigate the role of SDR9C7 in the ESCC metastasis, repeated transwell assays were adopted to establish highly and non-invasive ESCC sublines, and western blot showed that SDR9C7 expression was markedly higher in highly invasive cells compared with non-invasive ones. Down-regulation of SDR9C7 dramatically inhibited the metastatic abilities in vitro and in vivo, and repressed the expression of MMP11 in highly invasive cells, indicating that SDR9C7 promotes ESCC metastasis partly through regulation of MMP11, and might be a potential prognostic and therapeutic marker for ESCC patients.

## Introduction

Esophageal squamous cell carcinoma (ESCC) has been ranked as the sixth leading cause of cancer death worldwide [1]. Most patients with ESCC are diagnosed at an advanced stage with lymph node (LN) metastasis, subsequently resulting in a poor outcome [2]. The lymphatic system serves as the primary pathway for metastasis, which has been identified as a key prognostic factor for clinical outcome in ESCC patients [3]. Therefore, a better understanding of the gene expression involved in the development of LN metastasis may lead to therapeutic improvements for ESCC patients. The development of ESCC LN metastasis is regarded to arise from a multiple-step process including primary tumor formation, LN invasion, and distant metastasis. This process may be caused by the accumulation of genetic changes. An abnormal expression pattern of a single gene has been correlated with the metastasis in ESCC [4], [5], [6]. Our previous study demonstrated that the nuclear expression of twist promotes lymphatic metastasis in ESCC [7]. However, the diagnostic and prognostic biomarkers for ESCC metastasis remain obscure.

The gene expression profiling assay (GEP) is an important approach for identifying of individual molecules in the primary tumors at the time of diagnosis that are associated with LN metastasis. Differences in gene expression profiles have been identified in the primary tumors of oral squamous cell carcinoma [8], lung cancer [9] and cervical cancer [10] with and without LN metastasis, which has also been performed to evaluate the genetic signature of the primary tumors of esophageal adenocarcinoma patients with and without LN metastasis [11], and the expression patterns of primary ESCC and the matched metastatic LN has also been distinguished by GEP assay [12]. However, the differences in GEPs have not been indentified between primary ESCC tumors that were N_+_ and N_-_ tumors.

The aims of this study were to identify the LN metastasis-associated genes in primary ESCC tumors, using GEP analyses. The short chain dehydrogenase/reductase family 9C, member 7 (SDR9C7), was used for further study, because 2 transcripts of this novel gene were present 7 times more frequently in N_+_ compared with N- tumors. To investigate the role of SDR9C7 in the metastasis of ESCC, repeated transwell assays were used to establish highly and non-invasive ESCC sublines. Then, we determined the influence of lentivirus-mediated SDR9C7 siRNAs on the ESCC metastatic potential. Overall, these data not only discovered a prognostic gene expression profile, but also identified SDR9C7 as a critical marker for ESCC metastasis.

## Materials and Methods

### Tissue Samples

The primary surgical tissues from 3 ESCC tumors that were N_-_, and 3 patients with strong N_+_ tumors, were collected for GEP assays from December 2009 to May 2010 (Table 1). A total of 104 paraffin-embedded tumor tissues (average age, 59.5 years; range, 37–77 years; 77 male and 27 female) were obtained from ESCC patients who underwent surgery during from April 2007 to April 2009. All patients were treated with three-field esophagectomy with extended lymphadenectomy at Xijing Hospital without preoperative anticancer treatment. All tumor tissues and LN metastasis were histologically confirmed, and the TNM stage was assessed according to the 7th edition of the TNM classification by the AJCC. No patients died of causes other than ESCC. The follow-up examinations were conducted from the date of discharge until death or the deadline date (April 31, 2012). All participants have provided their written informed consents to participate in this study, and this study was approved by the ethics committees of Xijing Hospital.

**Table 1:** The clinical characteristics of patients included for gene expression profiling analysis.

Case	Gender	Age	TN stage	Differentiation	Location
1	Man	68	T3N0	Mederate	Middle
2	Man	59	T3N0	Well	Lower
3	Man	62	T4aN0	Poor	Middle
4	Man	63	T1bN3	Mederate	Middle
5	Man	53	T2N3	Well	Lower
6	Man	68	T2N3	Poor	Middle

### Gene Microarray and Data Acquisition

For GEP analysis, the total RNA from each sample was amplified and labeled by the Low RNA Input Linear Amplification kit (Agilent Technologies, Santa Clara, CA, USA), 5-(3-aminoallyl)-UTP (Ambion, Austin, TX, USA), and Cy3 NHS ester (GE Healthcare Biosciences, Pittsburgh, PA, USA) according to manufacturer’s protocol. The labeled cRNA was purified by the RNeasy mini kit (Qiagen, GmBH, Germany).

The kit was purchased from Agilent Technologies, Santa Clara, USA. Each slide was hybridized with 1.65 µg of Cy3-labeled cRNA using the Gene Expression Hybridization Kit in a hybridization oven. After 17 hours, the slides were washed in staining dishes (Thermo Shandon, Waltham, MA, USA) with the Gene Expression Wash Buffer Kit, and the stabilization and drying solution followed the manufacturer’s procedures. The samples were scanned by the Agilent Microarray Scanner and analyzed with the Feature Extraction software 10.7 using default settings. The raw data were normalized by Quantile Algorithm, Gene Spring Software 11.0 (Agilent Technologies, Santa Clara, CA, US).

### Immunohistochemistical Staining

Immunohistochemistical analyses were performed as previously described [13]. The sections were incubated with SDR9C7 antibody (Sigma, 1∶100), and sections were incubated with PBS in place of the primary antibody performed for control staining. The results were examined by microscopy by two independent pathologists blinded to the clinical data. The intensity was scored as 0, 1, 2 or 3 based on the staining intensity. The immunoreactivity proportion was ranked as 0 (0%), 1(0–30%), 2(30–60%) or 3(>60%) respectively. The two scores were added to obtain the final results: Negative (−), 0∼2; Positive (+), 3∼6.

### Highly and Non-invasive ESCC Sublines Construction

ESCC cell lines EC109 and EC9706 were purchased from the Chinese Academy of Medical Science (Beijing, China) [14] and were routinely maintained in our lab in 1640 medium (GIBCO, Carlsbad, CA) supplemented with 10% fetal bovine serum at 37°C in humidified air containing 5% carbon dioxide. Highly and non-invasive EC9706 and EC109 sublines were constructed using repeated transwell assays as described previously [15]. After a ten-round selection and expansion, the highly invasive EC9706 and EC109 sublines were established and designated as EC9706-P and EC109-P, and the non-invasive cell lines were named EC109-N and EC9706-N.

### Lentivirus-mediated siRNA Construction and Transfection

Lentivirus-mediated siRNAs with GFP were constructed by Shanghai Gene Chem Co, Ltd. The sequence for interfering with endogenous SDR9C7 expression was 5′-GCATGGAGCATGCTATTGTTT-3′, and the control Sequence (5′-CCAGAAGA GCAATCTGTAC-3′) targeting no known genes was used as a negative control. The SDR9C7 siRNA and control lentivirus were transfected into EC109-P and EC9706-P cells following the manufacturer’s protocol. Flow cytometry (FACScan; Becton Dickinson, San Jose, CA) was used to separate GFP-positive cells, and the purified cell lines were named Con-EC109-P, Si-EC109-P, Con-EC9706-P and Si-EC109-P.

### Protein Preparation and Western Blot Analyses

Protein preparation and western blot analyses were performed according to previously published protocols [13]. The cell proteins were prepared and separated on SDS-PAGE gels. The expression of β-actin was used as loading controls. The following antibodies were used as followings: anti-SDR9C7 (Abcam, 1∶500); anti-VEGF (Abcam, 1∶500); anti-E-cadherin(Santa, 1∶100); anti-MMP11(Cell Signaling Technology, 1∶300), and anti-β-actin (Sigma, 1∶4000).

### Proliferation Assay

The MTT assay was used to evaluate the proliferation of ESCC cell as previously described [13]. The absorbance values were determined by measuring the absorbance of the well at 490 nm using an ELISA reader (Bio-Rad Laboratories, CA). Each cell line was detected in triplicate.

### Migration and Invasion Assays

Cells migration and invasion assays were performed as described in previous study [16] using transwells (8-µl pore size, Corning, USA). After 3-washes by PBS and air-dried, cells were counted under a microscope at ×200 magnification on 3 random fields in each well. Each experimental condition was repeated in triplicate.

### Experimental Metastasis

The animal experimentation was performed according to the Institutional Animal Care and Use Committee guidelines of the Experiment Animal center of Fourth Military Medical University, and te approval ID as No 12015 by Experiment Animal Center of Fourth Military Medical University. Because EC9706-P cells demonstrated a more invasive phenotype in vitro, Con-EC9706-P and Si-EC9706-P cells were chosen for in vivo experiments with BALB/C-nu/nu nude mice (Shanghai Laboratory Animal Center of China) to induce metastases through caudal vein injection according to NIH Animal Care and Use Committee guidelines. Approximately 2×10^6^ cells of each cell line in 200 µl of medium without serum were injected into the nude mouse caudal tail vein. Each group contained 5 mice, which were maintained in a sterile animal facility for 7 weeks before being sacrificed. The mice were killed by the cervical dislocation method, and their lung and liver tissues were examined for metastases and also made into serial sections before HE staining for microscopic examination.

### Statistical Analyses

All statistical analyses were performed using SPSS 17.0. Student’s t-test was performed to analyze the results of gene expression profiling assays. The Kruskal–Wallis *U* or *H* test was used to analyze the significance of SDR9C7 expression as correlated with clinical factors, and the one-way ANOVA test was performed to evaluate the difference between three comparisons in cell proliferation, migration and invasion assays. The Kaplan-Meier method was used for univariate analysis, and a Cox regression model was used for multivariate analyses. A value of *P*<0.05 was considered significant.

## Results

### Identification of Differentially Expressed Genes

GEP assays were performed to identify the differentially expressed genes between the N_-_ and N_+_ primary ESCC tissues. The up-regulated or down-regulated transcripts with a false discovery rate (FDR) <0.01 and FCA absoluteare >4 are shown in Table 2 and 3. A total of 26 transcripts were increasingly expressed in N_+_ tumors to 23 different genes, and a total of 32 transcripts with decreased expression in N_+_ tumors correspond to 30 different genes (Fig. 1).

**Figure 1:** Gene expression profiling analysis of differential expression genes in ESCC with and without LN metastasis. Red color represents the up-regulated genes, and green or blue color represents the down-regulated genes in ESCC with LN metastasis. a, Hierarchical clustering analysis of genes associated with LN metastasis, N+, positive lymph node metastasis; N-, negative lymph node metastasis. b, Volcano plot analysis of differential expressed genes in ESCC between with and without LN metastasis. The x axis represents the differential expression profiles with the fold-induction ratios in a log2 scale, and the y axis represents the P value of T-test in a log10 scale.

**Table 2:** The probes of the up-regulated genes and their corresponding transcript names.

ProbeName	P-Value	Fold change	Gene Symbol
A_23_P134946	0.005	4.01	LRRC14
A_23_P219072	0.006	4.28	SAMD9
A_23_P355244	0.007	4.50	SAMD9
A_23_P259692	<0.001	4.96	PSAT1
A_24_P191047	0.008	5.69	CRCT1
A_23_P103617	0.006	5.85	ANXA9
A_23_P68487	0.005	5.89	BMP7
A_23_P127663	0.010	5.95	PRRG4
A_23_P11025	0.008	6.17	ZNF185
A_24_P332314	0.003	6.41	FAM111B
A_24_P91566	0.003	6.47	BMP7
A_23_P104522	0.007	7.04	NEBL
A_23_P17814	0.004	7.27	PLA2G3
A_23_P115478	0.006	7.31	PADI1
A_23_P8253	0.004	8.38	RAET1E
A_23_P25086	0.009	8.70	SDR9C7
A_23_P371758	0.009	9.32	SDR9C7
A_32_P154053	0.002	9.71	ATG9B
A_23_P254654	0.005	10.15	CLIC3
A_23_P76743	0.006	10.58	ASPG
A_32_P536872	0.003	12.40	TDRD5
A_23_P27473	0.002	13.35	CNFN
A_24_P76558	0.003	14.57	PLAC4
A_24_P236935	0.002	14.78	KLK6
A_24_P411515	<0.001	18.54	TMPRSS11F
A_23_P144417	<0.001	33.33	TMPRSS11D

**Table 3:** The probes of the down-regulated genes.

ProbeName	P-Value	Fold change	Gene Symbol
A_32_P217750	0.009	4.12	IL3RA
A_23_P434398	0.002	4.13	TXLNB
A_23_P72651	0.009	4.14	ECSCR
A_23_P315451	0.009	4.21	KIRREL2
A_23_P39237	0.009	4.27	ZFP36
A_23_P62115	0.001	4.45	TIMP1
A_23_P374695	0.003	4.66	TEK
A_24_P648880	0.003	4.80	MEIS3P1
A_24_P237328	0.007	4.87	MCAT
A_32_P100439	0.007	4.94	C7orf41
A_24_P945113	0.008	4.98	ACVRL1
A_32_P32413	0.009	4.99	SETBP1
A_23_P4551	0.003	5.19	SETBP1
A_23_P119196	0.009	5.29	KLF2
A_23_P315320	0.006	5.37	IL27
A_23_P212105	0.001	5.39	DAZL
A_23_P1083	<0.001	5.48	GJA4
A_23_P44244	0.009	5.92	SMARCA1
A_24_P185854	0.006	6.35	DMD
A_23_P329321	<0.001	6.56	PLB1
A_24_P412734	0.004	6.57	PRSS36
A_23_P121813	0.005	6.96	ENPP6
A_23_P38712	0.007	7.022	ADCYAP1
A_32_P47754	0.009	7.23	SLC2A14
A_24_P335781	0.009	7.25	ADCYAP1
A_24_P148907	0.008	7.27	MAB21L2
A_23_P140384	0.007	7.36	CTSG
A_32_P55871	0.008	10.08	C3orf15
A_23_P421436	0.004	11.46	ADD2
A_23_P33356	0.009	14.68	ADAMTS9
A_24_P97342	0.002	31.18	PROK2
A_23_P381505	<0.001	31.41	VWDE

### Up-regulated SDR9C7 Associated with Clinical Parameters

Two transcripts of the SDR9C7 gene were present 7 times more frequently in N_+_ tumors compared with N_-_ tumors, indicating that SDR9C7 might be a significant prognostic signature for ESCC metastasis. The expression of SDR9C7 was further detected in 104 ESCC tissues by immunohistochemical staining, and presented positive staining in the cytoplasm of ESCC tissues (Fig. 2a–d). The positive rate was 64.4%(67/104). The relationship between SDR9C7 expression and the patients’ clinicopathological data including gender, age, TNM stage, differentiation, lymphatic invasion and LN metastasis are presented in Table 4. Positive expression of SDR9C7 was significantly correlated with lymphatic invasion and LN metastasis (*P<*0.001). However, SDR9C7 expression had no significant correlation with age, sex, differentiation and T stage (Table 4; *P*>0.05).

**Figure 2:** Immunohistochemical staining of SDR9C7 expression in representative ESCC. The staining of SDR9C7 occurred in cytoplasm of cancer cells. a and b, ESCC tissues with lymph node metastasis; c and d, ESCC tissues without lymph node metastasis original magnification, (SP×200). e, Kaplan–Meier survival curves for patients with ESCC according to the expression of SDR9C7. The survival rate for patientswith positive SDR9C7 expression was significantly lower than that for patients with negative SDR9C7 expression (*P* = 0.001).

**Table 4:** SDR9C7 expression correlated with the clinical data of the patients.

Factor	Total	Negative	Positive	*P*-value
Age				0.54
≤59	52	20	32	
>59	52	17	35	
Gender				0.78
Men	77	28	49	
Women	27	9	18	
Location				0.19
Upper	28	6	22	
Middle	56	23	33	
Lower	20	8	12	
Differentiation				0.008
Well	49	23	26	
Moderate	39	10	29	
Poor	16	4	12	
Lymphatic invasion				<0.001
No	40	25	15	
Yes	64	12	52	
LN metastasis				<0.001
N0	50	31	19	
N1	35	6	29	
N2	17	0	17	
N3	2	0	2	
T stage				0.11
1	13	7	6	
2	42	18	24	
3	47	12	35	
4	2	0	2	

The associations of SDR9C7 expression with clinical factors were detected by Kruskal-Wallis *H* or *U* test.

### The Relationship between SDR9C7 Expression and Patient Prognosis

To further understand the clinical implications of SDR9C7 expression in ESCC patients, we analyzed the relationship between SDR9C7 expression levels and patient prognosis. The total survival rate of all patients with ESCC during the observation period was 41.3%. The mean follow-up time was 31.8 months with a median value of 24 months. The survival rate in patients with positive SDR9C7 expression was 29.9% (20/67), which was significantly lower that the survival rate in patients with negative SDR9C7 expression 62.2% (23/37). The Kaplan–Meier postoperative survival analyses showed that the following factors significantly correlated with postoperative survival: differentiation (*P* = 0.005), LN metastasis (*P*<0.001), lymphatic invasion (*P*<0.001), T stage (*P*<0.001) and SDR9C7 expression (Fig. 2 e; Table 5; *P* = 0.001). Multivariate regression analyses revealed that differentiation (*P* = 0.02), lymphatic invasion (*P* = 0.03) and T stage (*P* = 0.001) were independent prognostic factors, however, SDR9C7 expression was not an independent prognostic factor (Table 6; *P* = 0.31).

**Table 5:** Univariate analysis of prognostic factors.

Factor	n	Survivalrate	*P*-value
Age			0.37
≤59	52	44.2% (23/52)	
>59	52	38.5% (20/52)	
Gender			0.38
Men	77	44.2% (34/77)	
Women	27	33.3% (9/27)	
Location			0.61
Upper	28	35.7% (10/28)	
Middle	56	42.9% (24/56)	
Lower	20	45% (9/20)	
Differentiation			0.005
Well	49	55.1% (27/49)	
Moderate	39	35.9% (14/39)	
Poor	16	12.5% (2/16)	
Lymphatic invasion			<0.001
No	40	70.0% (28/40)	
Yes	64	23.4% (15/64)	
LN metastasis			<0.001
N0	50	64.0% (32/55)	
N1	35	28.6% (10/35)	
N2	17	5.9% (1/17)	
N3	2	0	
T stage			<0.001
1	13	76.9% (10/13)	
2	42	52.4% (22/42)	
3	47	23.4% (11/47)	
4	2	0	
SDR9C7			0.001
Negative	37	62.2% (23/37)	
Positive	67	29.9% (20/67)	

The univariate analysis reveals that differentiation, LN metastasis, lymphatic invasion, T stage and SDR9C7 expression significantly correlate with patient prognosis.

**Table 6:** Multivariate analysis of prognostic factors.

Features	95%CI	*P*-value
Age	0.63–1.83	0.80
Gender	0.43–1.32	0.32
Location	0.69–1.45	0.90
Differentiation	1.10–2.16	0.02
LN metastasis	0.80–1.86	0.35
Lymphatic invasion	1.08–5.72	0.03
T Stage	1.41–3.87	0.001
SDR9C7	0.71–3. 0	0.31

Multivariate analysis shows that differentiation, lymphatic invasion and T stage are significantly correlated with the patient prognosis.

### SDR9C7 Expression Correlated with Cell Invasive Potential

Repeated transwell assays were used to develop the highly invasive and the non-invasive ESCC cell lines. Statistical analyses showed that the levels of migration and invasion of the highly invasive cell lines EC109-P and EC9706-P were significantly stronger than the matched non-invasive cell lines EC109-N and EC9706-N (Fig. 3 a–b). The western blot analyses showed that SDR9C7 expression was markedly higher in EC109-P and EC9706-P cells compared with the matched non-invasive cell lines (Fig. 3c), indicating that SDR9C7 might be associated with the invasive phenotype of the ESCC cells.

**Figure 3:** Expression of SDR9C7 correlated with the invasive potential of ESCC cell lines. a and b, both migration and invasion assays showed that the migration and invasion ability of highly invasive ESCC cells were significantly higher than matched non-invasive cells. c, Western blot revealed that the expression of SDR9C7 was obviously higher in highly invasive ESCC cells compared with matched non-invasive cells. ^*^ Statistical significance (^a^ *P*<0.05 versus matched non-invasive cells).

### Knockdown of the SDR9C7 Inhibited ESCC Cell Metastasis in vitro

To identify the influence of SDR9C7 on ESCC proliferation, migration and invasion, lentivirus-mediated SDR9C7 siRNA and control siRNA were transfected into EC9706-P and EC109-P cells. Western blot analyses confirmed that SDR9C7 protein was significantly down-regulated by lentivirus-mediated SDR9C7 siRNA transfection in both EC109-P and EC9706-P cells (Fig. 4 a–b). As shown in Fig. 4 c and d, there was no significant difference in the growth rate between SDR9C7 knockdown cells compared with the controls (*P*>0.05). The results of the transwell assays showed that the migration and invasion of SDR9C7 siRNA-transfected EC109-P and EC9706-P cells were notably reduced compared with untreated cells or cells transfected with a control siRNA (Fig. 4 e–h). These results indicated that SDR9C7 overexpression played an important role in ESCC cell invasion in vitro.

**Figure 4:** Lentivirus-mediated siRNA targeting SDR9C7 Inhibited the metastasis of ESCC in vitro and in vivo. a and b, Western blot analysis showed that SDR9C7 expression was significantly down-regulated by lentivirus-mediated siRNA targeting SDR9C7 compared with mathced controls. β-actin was used as loading control. c and d, MTT showed that SDR9C7 knockdown couldn’t significantly influence the growth of ESCC cells. e and f, Repressing SDR9C7 expression decreased the migration and invasion of EC109-P cells. g and h, Inhibiting SDR9C7 decreased the migration and invasion of EC9706-P cells. i, Representative HE staining of lungs and livers isolated from mice that received injections of Con-EC9706-P or Si-EC9706-P cells. j, Incidence of metastasis in lungs and livers of mice. *Statistical significance (*P*<0.05, Si-EC109-P or Si-EC9706-P versus matched controls).

### Down-regulated SDR9C7 Inhibited ESCC Cell Metastasis in vivo

To further study the influence of SDR9C7 on ESCC metastasis in vivo, the highly invasive ESCC cells and the siRNA-transfected cells were used to induce experimental metastases in mice. Consistent with the in vitro results, the animal experiments showed that liver and lung metastases were apparently recognized in mice injected with Con-EC9706-P cells, but few metastases were observed in mice injected with SDR9C7-siRNA transfected cells (Fig. 4i). Histological analyses revealed that the number and the size of metastatic nodules in the lungs and livers of mice were significantly smaller in the controls (Fig. 4j; *P*<0.01). Thus, down regulated SDR9C7 inhibited the metastasis of ESCC in vivo.

### Molecular Mechanisms of SDR9C7 Involved in the Metastasis of ESCC

To explore the potential mechanisms of SDR9C7 involved in the metastasis of ESCC, we examined the expression of metastasis-related molecules, including MMP11, VEGF and E-cadherin, in highly invasive cells transfected with SDR9C7 siRNA and control lentivirus (Fig. 5). The results showed that inhibiting SDR9C7 expression can markedly repress the expression of MMP11, but no obvious alteration observed on VEGF or E-cadherin expression. These data indicated that SDR9C7 might influence ESCC cell metastasis partially through regulating MMP11 expression level. Moreover, other molecular mechanisms are supposed to be further studied in future work.

**Figure 5:** Effects of SDR9C7 siRNA on the expression of metastasis-related molecules by western blot analysis. The expression of MMP11 was markedly inhibited in cells transfected with siRNA compared with controls. β-actin was used as an internal control. The pictures shown are representatives of 3 independent experiments.

## Discussion

Lymphatic metastasis is a critical prognostic factor for the clinical outcome of ESCC patients, and may be involved in models of operation and chemotherapy program selection. The patients without lymphatic dissemination can benefit from a more limited transhiatal surgery or organ-preserving endoscopic resection, as opposed to these patients with lymphatic dissemination, who require a more extensive therapy. However, the methods for determining the status of LN metastasis including EUS, CT and PET/CT x-ray examination in ESCC patients are not always accurate. Interestingly, in our clinical work, we discovered that individuals showed a variable potential for lymphatic metastasis. Some T1 patients presented with a highly metastatic potential, but some T3 and T4 patients were found without lymphatic metastasis, which may be attributed to the gene expression signatures of the primary tumor tissues. Therefore, the identification of reliable molecular prognostic markers for LN metastasis of ESCC is critical for the improvement of therapeutic strategies for ESCC patients.

In the present study, we identified molecular prognostic markers for LN metastasis in primary ESCC tissues by gene expression microarray analyses. A total of 23 genes were found to reveal significantly higher expression levels, and 32 genes had significantly lower expression in N_+_ tumors compared with the N- ones. Of the 23 identified genes, a novel gene SDR9C7 is of particular interest because two transcripts of this gene were shown 7 times more frequently in N_+_ tissues compared with the N_-_ ones. In addition, we checked the protein expression of SDR9C7 in 104 paraffin-embedded ESCC tissues by immunohistochemical analyses. Our study showed that over-expression of SDR9C7 was associated with lymphatic invasion and LN metastasis in these ESCC patients. Univariate analyses showed that evaluation factors including poor differentiation, lymphatic invasion, LN metastasis, advanced T stage and SDR9C7 expression correlated with poor prognosis. However, those factors like age and gender exhibited no prognostic value.

SDR9C7, also named RDHS, SDR-O, a retinol dehydrogenase similar protein, was localized in 12q13.3, which was cloned in 2002 [17]. The SDR superfamily is one of the largest enzyme superfamilies with over 46,000 members in the sequence databases [18]. These enzymes were found to be involved in multiple physiological roles including steroid hormone, prostaglandin and retinoid metabolism and are therefore involved in signaling [19], and the metabolization of lipids and xenobiotics [20]. A growing number of single-nucleotide polymorphisms of SDR genes have been identified, and abnormalities of SDR genes cause a variety of inherited metabolic diseases [21]. SCDR10B was found to be up-regulated in human lung cancer [22]. As far as we have concerned, there is no reported data regarding SDR9C7 expression in human cancer. Therefore it is necessary to investigate the expression and the role of SDR9C7 expression in ESCCs.

To investigate the effects of SDR9C7 on ESCC metastasis, highly invasive and non-invasive EC109 and EC9706 cell subpopulations were constructed using a repeated transwell approach. Migration and invasion assays showed that the migration and invasion capabilities of EC109-P and EC9706-P cells were significantly stronger than the matched non-invasive cell lines, indicating that the cell models are suitable to study ESCC metastasis. Consistent with the results of the gene expression profiles, western blot analyses confirmed that the expression of SDR9C7 was significantly higher in the highly invasive lines compared with the matched non-invasion cells. Then lentivirus-mediated siRNA targeting SDR9C7 was transfected into EC109-P and EC9706-P cells. The MTT assays showed that SDR9C7 knockdown did not markedly influence the cell proliferation, but significantly inhibited the cell migration and invasion, indicating that SDR9C7 is an important factor for ESCC metastases. In addition, western blot assays revealed that inhibiting SDR9C7 expression could markedly repress the expression of MMP11, but not VEGF or E-cadherin. Thus, decreasing SDR9C7 repressed the metastasis of ESCC might be partially by regulating MMP11 expression.

In conclusion, for the first time, the present study identified LN metastasis-related genes by comparing the expression profiles of primary ESCC tumors with and without LN metastasis. Within our observation, SDR9C7 expression correlated with LN metastasis, lymphatic invasion and poor patient prognosis. Knockdown of SDR9C7 could significantly inhibit the metastasis of ESCC cells. These findings suggest that SDR9C7 plays an important role in the metastasis of ESCC. In addition, the present study provides valuable information for further exploration of identifying the molecular mechanisms of SDR9C7-involved ESCC metastasis.
